RETRACTED

# Diagnostic Value of Specialist Systems in Sports Knee Injuries

**DOI:** 10.1155/2022/1892877

**Published:** 2022-08-31

**Authors:** Xi Chen, Ao Yu, Ning Cai, Saite Wei, Yongqing Tong

**Affiliations:** ^1^College of Physical Education, Taiyuan University of Technology, Taiyuan, Shanxi 030000, China; ^2^Woosuk University, Jeonju, Republic of Korea

## Abstract

In order to explore the diagnostic effect of the expert system in knee sports injury, a method of diagnostic value of expert system in sports knee sports injury is proposed. This paper mainly takes 200 professional football players in sports higher vocational colleges as the research object. There are 146 male athletes and 44 female athletes; we establish a football injury ontology knowledge base and use a reasoning engine to build an intelligent expert system diagnosis system, allowing users to quickly discover diseases, accurately diagnose injuries, and obtain the best means of rehabilitation. Through the investigation, it can be seen that the body parts caused by football injuries are more complex, and the types of injuries in each part are also different. Therefore, it is particularly important to establish an intelligent retrieval system with convenient query and clear diagnosis by the expert system. With the birth and development of computer and artificial intelligence technology, the development of artificial intelligence expert systems in the medical field has become a reality. The construction of this system will have theoretical and practical significance and application value.

## 1. Introduction

Expert system (ES), also known as knowledge-based system, is the most important and successful field of artificial intelligence research. The expert system came into being in the mid-1960s. After more than 30 years of research and development, it is becoming more and more mature in theory and technology. It has been widely used in all fields all over the world and has achieved great economic and social benefits [1]. At present, the main application fields of expert system are as follows: medical diagnosis, chemical engineering, speech recognition, image processing, financial decision-making, signal interpretation, geological exploration, commercial decision-making, crop field management, farm management, petroleum, military, and so on. The expert system has become one of the research focuses of countries all over the world. Japan, the United States, Britain, and other countries have listed it as a national key research project and invested a lot of manpower and funds. Japan regards the expert system as the core content of the fifth-generation computer research, and Britain has listed the expert system/intelligent database as one of the four key research directions of the country [2]. The expert system is mainly composed of three parts (Figure 1): man-machine interface, knowledge base, and inference engine.

1. Man machine interface: the man machine interface, also known as man-machine interface, is the part where users communicate with expert system [3]. Through the man-machine interface, the user inputs the data and information required by the expert system. The system displays results and information through the man-machine interface. The media for users to communicate with the system can be text, sound, image, graphics, animation, audio-visual, etc. A friendly man-machine interface is one of the necessary conditions for a successful expert system, because it is the most direct part for users to communicate with the expert system. Its function and appearance are directly related to whether users can happily accept all the information transmitted by the system to them [4]
2. Knowledge base: used to store the expertise provided by domain experts. These expertise include book knowledge related to the field, common sense knowledge, and experience knowledge obtained by experts in practice. The problem solving of the expert system is carried out by using the special knowledge provided by experts to simulate the thinking mode of experts. Therefore, the quantity and quality of knowledge in the knowledge base have become the key factors of system performance and problem solving ability in an expert system. Therefore, the establishment of knowledge base is the central task of constructing expert system [5]
3. Reasoning machine: a program used to memorize the rules and control strategies adopted by the inference engine, so that the whole expert system can work in a logical way. Inference engine can use knowledge to reason and draw conclusions, rather than simply searching ready-made answers [6]
4. Interpretation facetyt: the interpreter can explain the behavior of the expert system to the user, including the correctness of the reasoning conclusion and the reason why the system outputs the candidate solution
5. Global database: also known as global database or general database, it is used to store the initial data of the field or problem and the intermediate data (information) obtained in the reasoning process, that is, some current facts of the processed object [7]

RETRACTED

## 2. Literature Review

He et al. believe that training without fatigue is ineffective and training without recovery is dangerous. However, it is also dangerous to exceed the maximum load of the knee joint. From the perspective of exercise physiology, after repeated overload stimulation of the knee joint for many times [8]. Chen et al. believe that the accumulation of fatigue and injury reduces the excitability of the nerve muscle contact, resulting in the disorder of the structure and metabolism of the internal dimension system of the joint, the fatigue of various tissues and cells, resulting in the abnormal energy metabolism and material metabolism of the whole knee joint, and the ability to maintain the movement of the knee joint can not be supplemented in time, resulting in the corresponding functional lesions of the knee joint [9]. Zhang believes that in the process of movement, the knee joint will produce corresponding compressive stress, tensile stress, shear stress, and hydrostatic pressure under various high-strength forces. In addition, there are reasons such as cartilage wear caused by mechanical stress imbalance or excessive load. The upper and lower bone levers of the knee joint are long, and the surrounding muscles are few. It is the most vulnerable joint in sports. The injury accounts for more than 50% in long jump. Athletes engaged in long jump have a history of acute or chronic injuries to varying degrees [10]. Meng et al. believe that in the standing long jump, consciousness dominates the body, and consciousness will be affected by psychological factors. In the long jump, psychological factors come from many aspects, which are mainly affected by the external environment and their own poor psychological quality. These two macrofactors are the main causes of sports injury to the knee joint [11]. Rudolph et al. believes that people's psychological development is slow and in the transition period from immature to mature, which will seriously affect the training process of athletes in the long jump and have a significant impact on the knee joint [12]. Li et al. believe that the knee joint is the link between the thigh and the lower leg. It is also the regulator that coordinates the up and down forces in the process of human movement and carries various internal and external factors such as gravity, self-generated gravity of the human body, and the supporting reaction force of the ground, so as to reduce the damage of human function in sports and play the role of dispersing pressure, transmitting weight, and reducing vibration. In this process, once the knee joint is overstimulated and the external force exceeds the maximum bearing capacity of the knee joint, violent injury will occur to the knee joint. At the same time, when excessive fatigue temporarily reduces the physical function, continuous long jump is also an important factor for acute injury [13]. Ren et al. believe that the repetitive injury of the knee joint is a closed cycle. Long-term single long jump exercise will make the knee repeatedly bear overload stimulation. With the increase of time, the accumulation of overload stimulation on the knee will produce fatigue wear on the knee. In the interval standing long jump training, although there will be an interval for the recovery of physical function in each long jump, it is the same exercise in a few hours, a day, a few days, or a few weeks [14]. Liu et al. believe that the main part of the movement is for the knee joint, which constantly repeats the flexion and extension of the leg and the indirect and repeated overload stimulation of various forces on the knee joint, which will reduce the muscle strength around the knee joint, reduce the proprioception, and reduce the range of joint movement, and the long-term sports injury or pathological sports injury will lose the sports ability of the knee joint [15]. Zhang et al. believe that in sports, knee injuries are more acute injuries, and acute injuries will turn into chronic injuries if they are not treated [16].

RETRACTED

Based on the current research, an expert system is proposed. This paper mainly takes 200 football professional athletes in sports vocational and technical college as the research object. There are 146 male athletes and 44 female athletes; we establish the ontology knowledge base of football injury and use the reasoning engine to build an intelligent expert system diagnosis system, so that users can quickly find the condition, accurately diagnose the injury, and get the best rehabilitation means.

## 3. Research Objects and Methods

### 3.1. Research Object

This paper mainly takes 200 football professional athletes in sports vocational and technical college as the research object. There are 146 male athletes and 44 female athletes.

### 3.2. Research Methods

1. Literature review method

By consulting relevant literature such as CNKI, this paper summarizes the various parts of football players that are easy to be injured in sports, as well as the direct or indirect factors that lead to injury in training and competition [17].

(2) Expert interview method

Through discussion with experts and professors in general hospital, sports medicine experts, and football coaches, it mainly focuses on the characteristics, clinical manifestations, and formation methods of sports injury related to football. During the interview with experts, many problems were put forward and discussed in depth and detail. The views and suggestions of experts were incorporated into the conclusions as a research basis [18].

(3) Questionnaire survey method

The necessity of constructing this system is analyzed in the form of a questionnaire. The specific implementation process and results are as follows: the questionnaire is mainly aimed at players, coaches, team doctors, bone and joint experts, and football administrators. The topics of the questionnaire are divided into three categories: closed, semiclosed, and open. Problems include common parts of football acute injury, common parts of football chronic injury, and common rehabilitation methods and prevention methods. Taking the sports vocational and technical college, the football field of the Provincial Sports Bureau, the Football Association, the provincial physical fitness Museum, the provincial hospital, and the orthopedic ward of the First Affiliated Hospital of Medical University as the distribution places, a total of 127 questionnaires were distributed, and 100 questionnaires were actually effectively recovered, with a recovery rate of 78.74%. This result can be used as the basis for the research results [19].

(4) This expert system has the characteristics of distributed processing

Its main purpose is to decompose the functions of a Ge family system and distribute them to multiple processors for parallel processing, so as to improve the processing efficiency of the system as a whole. It can work in a tight multiprocessor working environment or a loose computer network environment, so its overall structure largely depends on its hardware environment. To design and implement a distributed expert system, the following problems need to be solved:

1. Function distribution: that is, the functions or tasks of each part of the system decomposed are reasonably and evenly distributed to each processing node
2. Knowledge distribution: according to the function distribution, the knowledge is reasonably divided and distributed to each processing node. On the one hand, the redundancy of knowledge should be reduced as much as possible; on the other hand, the inconsistency of knowledge should be avoided as much as possible [20]
3. Interface design: the purpose of the interface design of each part is to make it easy for each part to communicate and synchronize with each other. On the premise of ensuring the completion of the overall task, it is necessary to make each part independent as far as possible, and the less the connection between parts, the better
4. System structure: the design of the system structure depends on the environment and nature of the application on the one hand, and the hardware environment on the other hand

Distributed artificial intelligence mainly studies how multiple intelligent systems dispersed logically or physically solve problems in parallel and cooperate with each other. The cognitive model of distributed artificial intelligence research is that most of human activities involve social groups, and the solution of large and complex problems needs the cooperation of multiple professionals or organizations. Distributed artificial intelligence theory has high application value in parallel programming, computer communication, network management, and control [21]. The main advantages of distributed expert system are as follows:

- It can effectively improve the problem-solving ability of the system. Firstly, the openness of the system is enhanced, and the problem-solving ability of the system can be improved by adding new logic processing nodes. In addition, due to the redundancy of communication path, processing node and knowledge, the system can still continue to operate in case of failure (allowing the reduction of response time or solution accuracy), and the reliability of the system is good
- It can effectively improve the efficiency of problem solving. Each node in the system can work in parallel, so it can scientifically allocate the tasks of each node, so that each node can solve the problem in a coordinated, parallel and fast manner at the same time, that is, use the distributed structure for parallel and efficient reasoning and calculation [22]
- It can effectively reduce the complexity of software. The system decomposes the solving task of the whole system into several relatively independent special subtasks, which reduces the complexity of the problem solving of each processing node

The research frontier of the distributed expert system is the research of distributed artificial intelligence based on multiagent structure, as well as the research of flexible and intelligent distributed software structure system, such as the research and construction of distributed computing architecture based on cD0M and CORBA technology.

RETRACTED

## 4. Research Results and Analysis

### 4.1. Results

The following results are obtained after the research according to the above methods, and the data are sorted and analyzed:

It can be seen from Figure 2 that the common injured parts of football sports include the knee, ankle, head, and foot, mainly ankle and knee joint injuries. Especially in high-intensity professional football matches, players are often very focused in the game, which is very easy to cause injury in physical confrontation. If the nonball player tackles the ball player, it will cause injury to the ankle and knee joint [23].

It can be seen from Figure 3 that among the common injuries in football sports, the main injury diseases of knee joint injury are cruciate ligament injury, medial ligament injury, lateral ligament injury, and meniscus injury. There are many ligaments in the knee joint, so there is a great possibility of strain and long recovery time. Therefore, offsite preparation activities should be sufficient and physical training should be scientific. In knee ligament strain, the most common cause of avulsion is that the knee joint is impacted by external force during torsion, and it is easy to cause osteoarthritis due to the knee joint with imperfect function of anterior cruciate ligament [24].

It can be seen from Figure 4 that among the common injuries in football, the injury rate of ankle sprain and contusion is the highest, followed by football ankle and ankle fracture. Because football players often jump to compete for the header, it is easy for two players to lose their center of gravity and land unsteadily due to fierce collision when taking off, which is very easy to cause ankle fracture. Through the investigation, we can see that the body parts caused by football injury are more complex, and the types of injuries in each part are also different. Therefore, it is particularly important to establish an intelligent retrieval system with convenient query and clear expert system diagnosis [25].

### 4.2. Establish Expert System Diagnosis Intelligent Retrieval System

1. Football injury information management query module

The system extracts keywords according to the damage location name or fuzzy representation selected by the user and retrieves the damage instance and corresponding attributes in the damage ontology database. The ER relationship diagram of this module is shown in Figure 5.

(2) Diagnosis module of football injury expert system

The system can judge through the user's selection or fuzzy input of the damaged part of the human body, and then through the selection of clinical manifestations, the system finally makes reasoning and judgment and feeds back the damage results diagnosed by the expert system to the user. The ER relationship diagram of this module is shown in Figure 6.

(3) Injury and rehabilitation means module

According to the injury inquired by the user, the system matches the reasonable rehabilitation treatment means mainly through the acute and chronic injury and feeds back to the user [26].

(4) The overall structure of the system is designed, and the specific expert system diagnosis flow chart is shown in Figure 7.

## 5. Conclusion

This paper chooses football injury as the research object. By extracting the field knowledge of football injury, constructing the ontology database, using the reasoning mechanism to realize the reasoning expert system diagnosis, and establishing the intelligent expert system diagnosis system, the system not only provides a useful exploration for the expert system diagnosis of football injury but also makes a contribution to the intelligent digital medical treatment. The main work is as follows:

1. The professional knowledge of football injury was extracted and discussed and verified with human experts. Then, the formal language is used to describe the knowledge and construct the ontology knowledge base
2. Add constraints to related classes in ontology knowledge base and realize internal retrieval through the built-in inference engine of Protégé tool
3. Jena inference engine is selected as the inference engine of the system, and its inference mechanism is used to complete the diagnosis of the inference expert system. The research results promote the innovation of the accuracy of knowledge expression in the field of football injury, the scientificity of organization construction, and the integrity of hierarchical structure and lay a solid foundation for improving the level of sports injury intelligent expert system diagnosis and establishing football injury disease database. It also lays a foundation for establishing a richer sports injury knowledge base and medical expert system diagnosis system in the future

RETRACTED

## Figures and Tables

**Figure 1:** Structure of an ideal expert system.

**Figure 2:** Proportion of common injury sites in football events (*n* = 200).

**Figure 3:** Proportion of knee joint injury diseases in football events (*n* = 200).

**Figure 4:** Proportion of knee joint injury diseases in football events (*n* = 200).

**Figure 5:** ER diagram of information management inquiry module of football injury.

**Figure 6:** ER diagram of football injury diagnosis module.

**Figure 7:** System framework diagram.

## Data Availability

The data used to support the findings of this study are available from the corresponding author upon request.
